This article has been retracted.

# Association of Single Nucleotide Polymorphism rs17580 with Smoking and Pulmonary Tuberculosis

**DOI:** 10.1155/2022/6984403

**Published:** 2022-04-09

**Authors:** Tao Li, Shunli Han

**Affiliations:** Pulmonary Department, Central Hospital of Jiaozuo Coal Industry (Group) Co., Ltd., Jiaozuo 454000, China

## Abstract

This study aimed to investigate the correlation between SERPINA1 single nucleotide polymorphism (SNP) rs17580, smoking, and pulmonary tuberculosis (TB). A total of 420 TB patients (observation group) and 640 patients without pulmonary disease (control group) were randomly included. The frequencies of different genotypes were counted in both groups, and the correlation between SNP genotypes and the occurrence of TB was analyzed. Statistical models were performed to analyze the correlation between rs17580 and TB and the correlation between rs17580. The frequencies of genotypes TT, TA, and AA at the rs17580 locus in patients with TB were not statistically different from those in the control group (*P* > 0.05), and the distributions of the two groups were in accordance with the Hardy–Weinberg equilibrium law. rs17580 was analyzed in dominant, recessive, and codominant models, exhibiting no statistical difference (*P* > 0.05). There was no significant difference among the three genotypes in the 1–5 typing (*χ*^2^ = 1.034, *P*=0.998), and the difference between T and C was not statistically significant (*χ*^2^ = 0.012, *P*=0.999). There was a significant difference between the three genotypes between the smoking group and the nonsmoking group in TB patients (*P* < 0.05). There was no significant difference among three genotypes in the alcoholic group and the nonalcoholic group in TB patients (*P* > 0.05). There was no statistical difference in the time to cure among the 3 genotypes in TB patients (*P* > 0.05). A type mutation of rs17580 in the SERPINA1 gene was strongly associated with a higher risk of development of TB in smoking patients.

## 1. Introduction

Pulmonary tuberculosis (TB) is an infection with a high incidence, which is affected by time or age [1], and is a common challenge for human health [2]. Tuberculosis is a bacterial disease caused by *Mycobacterium tuberculosis*, which is mostly transmitted through the respiratory tract and closely related to the health status of the host. If the host organism has a reduced ability to clear and limit infection with *Mycobacterium tuberculosis*, it is highly susceptible to infection with the bacteria. It has been suggested that lifestyles, work environment, and outdoor air quality may have a certain impact on the health of the host [3, 4], especially smoking and passive smoking in a closed environment can not only reduce the resistance of the respiratory organs, making it easy for harmful microorganisms such as *Mycobacterium tuberculosis* to invade the lungs and make tuberculosis more likely to occur, causing bacteria or viruses infection while the resistance of the respiratory organs is further reduced, making TB more difficult to cure [5, 6]. Studies have found that differences in human genetic polymorphisms may lead to differential susceptibility to TB [7], and susceptible individuals must pay more attention to lung protection and screening.

SERPINA1 encodes *α*-1-antitrypsin, which complexes with and inhibits the activity of neutrophil elastase, produced primarily by hepatocytes, monocytes, alveolar macrophages, enterocytes, and myeloid cells. Subjects with variants in one or both copies of the SERPINA1 gene may develop *α*-1-antitrypsin deficiency and are at risk for emphysema and/or chronic liver disease because elastase activity in the lung and liver is greater than normal [8, 9]. The base T mutation to A in rs17580, which is located in the coding region of the SERPINA1 gene, causes a change in amino acid from glutamate to valine, which alters the entire protein structure and affects the function of the encoding enzyme [10, 11]. Studies have found that the occurrence of drug resistance of *Mycobacterium tuberculosis* is related to mutations of multiple genes [12, 13]. A recent study found a high correlation between mutations in the SERPINA1 gene and chronic obstructive pulmonary disease [14]. The effect of this gene on lung disease is mostly reflected by levels of gene expression [15, 16] and has not been analyzed in terms of gene polymorphism. Since differences in genetic polymorphisms make humans differently susceptible to *Mycobacterium tuberculosis*, it is necessary to further explore the effect of genetic polymorphisms on *Mycobacterium tuberculosis* susceptibility. The rs17580 is a single nucleotide polymorphic locus on the SERPINA1 gene, which is located in the coding region of the SERPINA1 gene, and mutations at this locus cause downregulation of gene expression and decrease the expression of the SERPINA1 gene in vivo, which can increase the risk of chronic lung disease [8, 11]. The aim of this study was to investigate the correlation between SERPINA1 SNP rs17580, smoking and the development of TB.

## 2. Materials and Methods

### 2.1. General Data

Patients (local residents, ethnic Han) with TB treated in our hospital from April 2015 to April 2017 were included according to the following criteria: (1) conforming to the diagnosis criteria of pulmonary tuberculosis WS 288–2017 (China); (2) positive sputum smear test; and (3) all patients were local residents, ethnic Han, and were diagnosed as tuberculosis in our hospital for the first time. The exclusion criteria were as follows: (1) TB with other comorbidities; (2) abnormal heart, liver, and kidney function; (3) diabetes mellitus; (4) women during pregnancy and lactation; and (5) patients with mental abnormalities. A total of 420 cases with TB were randomly included in the observation group, and another 640 patients without pulmonary disease who came to our hospital were also randomly enrolled as the control group. The observation group had 240 males and 180 females, aged 29–83 years, with an average of (55.2 ± 17.3) years, and the control group had 380 males and 260 females, aged 27–82 years, with an average of (53.8 ± 19.3) years. All patients were informed about the study and signed the informed consent form, which was approved by the ethics committee of Central Hospital of Jiaozuo Coal Industry (Group) Co., Ltd.

### 2.2. Methods

#### 2.2.1. Extraction of Genomic DNA

Extraction of genomic DNA was performed as previously described [17]. 5 mL of whole blood was collected from each patient using an anticoagulation tube containing Edathamil (EDTA-K2). Genomic DNA of blood was extracted using the Omega Mag-Binds Forensic DNA Kit (OMEGA, Doraville, GA, USA), and the concentration and purity of DNA were determined by nanodrop and stored at −20°C.

#### 2.2.2. PCR for SNP Typing

PCR was applied for SNP typing [17]. The primer sequences and their Taqman probe sequences at the SNP sites were designed using Oligo 6.0 (Table 1), and primer synthesis was done by Shanghai Biotech (Shanghai, China). 1 *μ*L of DNA solution and 1.2 *μ*L of primer solution (0.4 *μ*L of upstream and downstream primers and probe primers) were added to 17.8 *μ*L of preconfigured TransStart Probe qPCR SuperMix (Beijing Quan-Shi Jin Biological Company, Beijing, China), mixed by slight shaking, and put into a Bio-Rad CFX96 fluorescence qPCR instrument with the reaction conditions in Table 2. The experimental results were generated by the instrument software. Three replicate wells were made for each sample, and DEPC water was used for the negative control, and a positive plasmid containing the sequence (synthesized by Bio-Rad Shanghai, Shanghai, China) was used for the positive control.

### 2.3. Statistical Analysis

Statistical analysis was performed using Statistical Product and Service Solutions (SPSS) 19.0 (SPSS Inc., Chicago, IL, USA) [18]. Lifestyle habits (including smoking and alcohol consumption) and TB genotypes were variables. The distribution of genotypes between observation and control groups as analyzed by a chi-square test. The relationship between each genotype and the risk of tuberculosis was analyzed by logistic regression, and Bonferroni correction was performed for pairwise comparisons between multiple samples, with *P* < 0.05 being a statistically significant difference.

## 3. Results

### 3.1. Baseline Data

There were no statistically significant differences between the two groups in terms of gender, age, and smoking and alcohol consumption (*P* > 0.05), as shown in Table 3.

### 3.2. Distribution of rs17580 Genotypes

The genotypes were determined as follows: the horizontal coordinate near FAM was wild pure, the vertical coordinate near HEX was mutation pure, and the position near the 45° line was heterozygous. Genotyping results were obtained in all patients (Figure 1). The distribution frequencies of genotypes TT, TA, and AA at the rs17580 locus in the TB patient group were not statistically different from those in the control group (*P* > 0.05; Table 4). The distribution of rs17580 genotypes was in accordance with the Hardy–Weinberg equilibrium law, P (control) = 0.42 and P (observation) = 0.43.

### 3.3. Analysis of the Risk of Tuberculosis

The three genotype models showed no significant differences in terms of the risk of tuberculosis. (*P* > 0.05; Table 5).

### 3.4. Correlation between Genotypes of rs17580 and TB Typing

The difference between the 3 genotypes in the 5 types of TB was not statistically significant (*χ*^2^ = 1.034, *P*=0.998), and the difference between T and C was not statistically significant (*χ*^2^ = 0.012, *P*=0.999) (Table 6).

### 3.5. Correlation between the Genotype of rs17580 Combined with Smoking and TB

There was a statistically significant difference (*P* < 0.05) between three genotypes between the smoking group and the nonsmoking group in patients with TB (Table 7).

### 3.6. Correlation between the Genotype of rs17580 Combined with Alcohol Consumption and TB

There was no statistical difference (*P* > 0.05) between three genotypes between the alcoholic group and the nonalcoholic group in patients with TB (Table 8).

### 3.7. Correlation between the Genotype of rs17580 and the Time to Cure in Patients with TB

There was no statistical difference in the time to cure among the three genotypes in patients with TB (*P* > 0.05) (Table 9).

## 4. Discussion

The harm of smoking to the lungs is obvious, and smoking is found in more than 80% of lung cancer patients, which is one of the most crucial factors triggering lung cancer [19]. Although smoking is harmful to the lungs, as a single factor, it does not have an effect on the incidence of tuberculosis, which was evidenced by the difference between the observation group and the control group.

Katoto et al. [20] concluded with several methods of SNP typing that the Taqman probe method has an irreplaceable advantage in correct typing. In this study, better genotyping results were obtained in all patients with TB and controls using this method. Do Linh San et al. [21] described that the A/T of rs17580 is highly associated with TB in European whites. However, we found that the mutant genotype of rs17580 was not significantly associated with the risk of tuberculosis in the group of the Chinese Han population. Also, no statistically significant association was found between mutations at this locus and typing in relation to the 5 subtypes of TB. It is possible that SNP mutations in the SERPINA1 gene do not affect tuberculosis in the same way among different ethnic groups, and therefore the correlation between base mutations and tuberculosis needs to be analyzed for different populations [22]. The result of the correlation between SNP and TB also varies depending on the sample size, so the larger the sample size, the more meaningful it is [23, 24]. However, those with mutations at this locus in the population with smoking habits were more likely to develop TB. This suggests that the gene may be more susceptible to the effects of substances in cigarettes, making the lungs more susceptible to infection with *Mycobacterium tuberculosis*, leading to the development of tuberculosis.

In conclusion, smoking patients with the A mutation in rs17580 of the SERPINA1 gene are strongly associated with the occurrence of tuberculosis.

## Figures and Tables

**Figure 1:** Typing results of rs17580. Near the *X*-axis is TT type, near the *Y*-axis is AA type, and the middle green part is TA type.

**Table 1:** Primer sequences.

SNP	Primer sequences	Probe sequences
rs17580	Upstream: 5′-TGGCTAAGAGGTGTGGGCAGC-3′	FAM: 5′-GTTCATTTTCCAGGTGCTG-3′
	Downstream: 5′-GATGAAATACCTGGGCAATGCC-3′	VIC: 5′-GTTCATTTACCAGGTGCTG-3′

**Table 2:** Condition procedure of PCR reaction.

Step	Temperature	Time	Cycle
1	94°C	3 min	1
2	94°C	15 s	42
	60°C	60 s	
	Read		

**Table 3:** Baseline data.

Parameters	Observation group (*n* = 420)	Control group (*n* = 640)	*P* value
Age (years)	55.2 ± 17.3	53.8 ± 193	0.484
*Sex*			
Male	240 (57.1%)	380 (59.4%)	0.733
Female	180 (42.9%)	260 (40.6%)	
BMI (kg/m^2^)	24.5 ± 1.6	24.6 ± 1.8	0.554
*Smoking*			
Yes	172 (41%)	274 (42.8%)	0.415
No	248 (59%)	366 (57.2%)	
*Alcohol addiction*			
Yes	242 (57.6%)	383 (59.7%)	0.536
No	178 (42.4%)	258 (40.3%)	

BMI: body mass index.

**Table 4:** Frequency distribution of rs17580 (*n*, %).

Genotype	Observation group (*N* = 420)		Control group (*N* = 640)		*χ* ^2^	*P*
	*N*	%	*N*	%		
TT	250	59.5	392	61.25	0.064	0.800
TA	128	30.5	216	33.75	0.242	0.623
AA	42	10	32	5	1.802	0.179
T	628	74.8	1032	80.6	0.971	0.324
A	212	25.2	248	19.4		

**Table 5:** Different models to analyze the risk of tuberculosis.

Model type	Genotype	Observation group (*N* = 420)	Control group (*N* = 640)	OR value ^(95% Cl)^	*P*
Dominant model	TT	250	392	1	0.800
	TA + AA	170	248	1.075 (0.745 to 1.553)	
Recessive model	TT + TA	378	608	1	0.179
	AA	42	32	2.111 (1.042 to 4.456)	
Codominant model	TT	250	392	1	0.395
	TA	128	216	0.929 (0.557 to 1.314)	
	AA	42	32	2.058 (0.855 to 4.548)	

OR: odds ratio.

**Table 6:** Distribution of genotypes of rs17580 in TB patients (*n*, %).

Typing	*N* (420)	rs17580				
		TT (*N* = 250)	TA (*N* = 128)	AA (*N* = 42)	T (*N* = 628)	A (*N* = 212)
Type I	72	42 (16.8)	24 (18.8)	6 (14.3)	108 (17.2)	36 (17)
Type II	96	58 (23.2)	28 (21.9)	10 (23.8)	144 (22.9)	48 (22.6)
Type III	82	48 (19.2)	26 (20.3)	8 (19)	122 (19.4)	42 (19.8)
Type IV	90	54 (21.6)	26 (20.3)	10 (23.8)	134 (21.3)	46 (21.7)
Type V	80	48 (19.2)	24 (18.8)	8 (19)	120(19.1)	40(18.9)

**Table 7:** The correlation between rs17580, smoking with the occurrence of tuberculosis (*n*, %).

Group	TT (*N* = 250)	TA (*N* = 128)	AA (*N* = 42)	T (*N* = 628)	A (*N* = 212)
Smoking (*N* = 172)	65 (37.8)	78 (45.3)	29 (16.9)	208 (60.6)	136 (39.4)
Nonsmoking (*N* = 248)	185 (74.6)	50 (20.2)	13 (5.2)	420 (84.7)	76 (15.3)
*χ* ^2^	27.508	14.303	6.964	14.615	
*P*	0.000	0.000	0.008	0.000	

**Table 8:** Correlation between rs17580, alcohol consumption with the occurrence of tuberculosis (*n*, %).

Group	TT (*N* = 250)	TA (*N* = 128)	AA (*N* = 42)	T (*N* = 628)	A (*N* = 212)
Alcohol addiction (*N* = 242)	134 (53.4)	82 (33.9)	26 (10.7)	350 (72.3)	134 (27.7)
Not addicted to alcohol (*N* = 178)	116 (65.2)	46 (25.8)	16 (9.0)	278 (78.1)	78 (21.9)
*χ* ^2^	2.62	1.567	0.163	0.902	
*P*	0.106	0.211	0.686	0.342	

**Table 9:** Correlation analysis between genotype of rs17580 and time to cure in patients with TB (*n*, %).

Group	TT (*N* = 250)	TA (*N* = 128)	AA (*N* = 42)	T (*N* = 628)	A (*N* = 212)
≤7 days (121)	67 (53.4)	41 (33.9)	13 (10.7)	175 (72.3)	67 (27.7)
>7 days (299)	183 (61.2)	87 (29.1)	29 (9.7)	453 (75.8)	145 (24.2)
*χ* ^2^	2.65	1.678	0.187	0.897	
*P*	0.116	0.234	0.732	0.421	

## Data Availability

The datasets used and analyzed during the current study are available from the corresponding author on reasonable request.
